# Aerial imagery reveals abnormal stingrays, *Taeniura lymma* (Myliobatiformes: Dasyatidae), in the central Red Sea

**DOI:** 10.1002/ece3.11399

**Published:** 2024-05-30

**Authors:** Ioana Andreea Ciocănaru, Brian Owain Nieuwenhuis, Raquel Lubambo Ostrovski, Jesse Cochran, Burton H. Jones

**Affiliations:** ^1^ Marine Science Program, Biological, Environmental Sciences and Engineering Division King Abdullah University of Science and Technology (KAUST) Thuwal Saudi Arabia; ^2^ Red Sea Research Center King Abdullah University of Science and Technology (KAUST) Thuwal Saudi Arabia

**Keywords:** bluespotted ribbontail ray, drone, incomplete disk closure, pectoral fin, symmetrical deformity

## Abstract

While morphological abnormalities have been widely reported in batomorphs, ontogenetic deformities of the posterior pectoral fin are rare. In this paper, we present two individuals of the bluespotted ribbontail ray, *Taeniura lymma* (Forsskål, 1775), with symmetrically deformed posterior pectoral fins. Both individuals were observed through aerial imagery on a coastal sandflat in the central Red Sea (22.30° N, 39.09° E). The similarity of this symmetrical deformity in both individuals indicates it likely has a genetic base. However, lacking access to the specimens, the ultimate cause of the abnormality remains uncertain. The incomplete disk closure did not seem to affect survival, as both individuals had reached a disk width of 22 cm, well above the typical birth size of the species. Our observations constitute both the first report of a morphological abnormality in *T. lymma* and the first record of a batomorph with a symmetrically deformed posterior pectoral fin.

## Graphical abstract

In this paper, we present two individuals of the bluespotted ribbontail ray, Taeniura lymma (Forsskål, 1775), with symmetrically deformed posterior pectoral fins. Both individuals were observed through aerial imagery on a coastal sandflat in the central Red Sea (22.30° N, 39.09° E). Our observations constitute the first report of a morphological abnormality in T. lymma.

## 1 INTRODUCTION

Morphological defects in batomorphs have been reported for over 130 years (Bureau, 1889), encompassing a wide range of deformities including misshapen genitalia, dental abnormalities, hermaphroditism, bicephaly, anophthalmia, albinism, and fin defects (Ehemann et al., 2022; Ribeiro‐Prado et al., 2008). Reports of fin deformities include the absence of fins (Capape et al., 2015; Ehemann et al., 2022), the presence of aberrant fins (Ben Brahim & Capapé, 1997; Deli Antoni et al., 2012), and deformed pectoral disk (Ramaiyan & Sivakumar, 1988; Ribeiro‐Prado et al., 2008; Valderrama‐Herrera et al., 2022). Anterior incomplete disk closure, in which the pectoral fins failed to completely fuse with the head, is the most commonly reported defect (Ehemann et al., 2022; Ribeiro‐Prado et al., 2008; Valderrama‐Herrera et al., 2022). Malformations along the posterior side of the pectoral disk are much rarer, but completely cleft posterior pectoral fins with a fringe‐like appearance have been reported in *Pateobatis jenkinsii* (Annandale, 1909) and *Dasyatis hypostigma* Santos & Carvalho, 2004 (Ramaiyan & Sivakumar, 1988; Ribeiro‐Prado et al., 2008).

The bluespotted ribbontail ray *Taeniura lymma* (Forsskål, 1775) is a small, benthic batomorph that is easily recognizable by its greenish–brown coloration punctuated with bright blue spots and tail stripes (Surapaneni et al., 2023). It is broadly distributed throughout the Indo‐Pacific and is generally associated with shallow coral reefs and adjacent habitats (Dabruzzi et al., 2013; Last et al., 2016). Juveniles tend to nurse in extremely shallow waters, including intertidal zones and other nearshore habitats (Dabruzzi et al., 2013; Leurs et al., 2023; O'Shea et al., 2012). Despite being common and broadly distributed in easily accessible habitats, *T. lymma* is poorly studied. This is likely due to the lack of conservation concern (Sherman et al., 2021). Here, we report the first observations of incomplete disk closure in two specimens of this species, and the first instance of a symmetrically deformed posterior pectoral disk in any batomorph.

## 2 METHODS

### 2.1 Study area

Abnormal bluespotted ribbontail rays were encountered by chance while inspecting Unoccupied Aerial Vehicle (UAV) imagery collected to monitor mangroves. All UAV surveys were conducted over a small *Avicennia marina* (Forssk.) Vierh. mangrove stand (~12,000 m^2^) within the campus of the King Abdullah University of Science and Technology (KAUST) on the Saudi‐Arabian coast of the central Red Sea (22.30° N, 39.09° E) (Figure 1). While centered on the mangrove fringe the UAV surveys included a part of the adjacent sandflat, which is where the bluespotted ribbontail rays were spotted. The depth of this sandflat ranges from 10 to 40 cm, and it is bordered by a deeper shipping channel (Figure 1a). Nearby sandflats (<2 km) were previously shown to harbor four batomorph species, with *T. lymma* being the most common (McIvor et al., 2022).

**FIGURE 1:** (a) ESRI World Imagery showing KAUST campus and surrounding reefs. White square indicates the study area, inset shows general location in the central Red Sea. (b) UAV orthomosaic of the study area showing the locations where deformed rays were sighted.

### 2.2 UAV surveys

Four aerial surveys were conducted, on February 8, February 23, April 8, and December 15, 2022. UAV surveys were conducted in the morning between 8 and 10 a.m. to minimize sun glint (Joyce et al., 2019). We used a DJI Matrice 300 RTK equipped with a 45‐megapixel, full‐frame DJI Zenmuse P1 camera with a DJI DL 35 mm F2.8 LS ASPH lens (DJI, 2021). The surveys were designed in the DJI Pilot 2 application and consisted of a lawn mower pattern at 20‐m altitude above ground/water level (AGL) with 80% frontal overlap and 75% side overlap. The horizontal speed of the UAV was 5.5 m/s, so a single survey was completed in approximately 15 min.

### 2.3 Ray detection and measurements

The 4110 images captured over the four flights were visually inspected for the presence of rays in the order of their acquisition. The high spatial resolution of our camera, the low flight altitude, and shallow study area allowed easy detection of rays. Additionally, the images from each flight were processed in Agisoft Metashape Professional to generate orthomosaics (Agisoft LLC, 2016; Casella et al., 2017). The orthomosaics were then used to plot the location of all ray detections. This allowed us to filter out duplicate detections of the same individual in parallel UAV transects. To measure each ray, we selected the image where the ray was close to the center of the frame (to minimize optical distortion caused by refraction) and its body or tail was not folded (for accuracy of measurement). The best image was loaded in the software FIJI, where disk width (DW) and total length (TL) were measured (Schindelin et al., 2012). The obtained pixel values were converted to standard linear units by multiplication with the Ground Sampling Distance, which was 0.25 cm/pixel (Equation 1) (DJI, 2021).

(1) $$\text{Ground Sampling Distance}=\frac{\text{Sensor width}\;\left(\mathrm{mm}\right)\times \text{Flight altitude}\;\left(m\;\mathrm{AGL}\right)}{\text{Focal length}\;\left(\mathrm{mm}\right)\times \text{Image width}\;\left(\text{pixels}\right)}$$

## 3 RESULTS

On February 23, 2022, we observed two individuals of *T. lymma* (Forsskål, 1775) with symmetrically deformed pectoral fins (Figures 1b and 2). Instead of the rounded disk typical for this species, the pectoral fin of these specimens made a straight cut toward the animal's centerline at approximately three‐quarters of the normal disk length (Figure 2). In the posterior quarter, only a small pointy lobe was present, allowing an unobstructed view of the pelvic fins from above. The two specimens can be distinguished based on their pelvic fins, which have a slightly unusual shape in Specimen 2 (Figure 2b). In Specimen 1, claspers appear to be visible, potentially indicating this is a mature male (Figure 2a). However, we cannot discount the possibility that what appears to be claspers is an unusual lobe of the pelvic fin in this already deformed individual. No clasper‐like structures are visible for the second specimen (Figure 2b). The deformed specimens were of similar size, both had a disk width of 22 cm and total lengths of 49 cm (Specimen 1) and 48 cm (Specimen 2). The size of the deformed rays falls neatly within the size range of the non‐deformed *T. lymma* specimens we observed in the area which had an average disk width of 21.7 cm (SD = 3.5, *n* = 24) and an average total length of 51.6 cm (SD = 11.3, *n* = 24) (Figure 3).

**FIGURE 2:** UAV images of *Taeniura lymma* specimens seen during our surveys. (a) Deformed specimen one seen on February 23, 2022. (b) Deformed specimen two seen on February 23, 2022. (c) The deformed specimen seen on April 8, 2022. This observation is thought to be a “recapture” of the specimen in panel (a). (d) A typical specimen seen on February 23, 2022.

**FIGURE 3:** (a) Disk width and (b) total length of the abnormal and normal rays observed during the UAV surveys.

On April 8, 2022, another observation of a deformed bluespotted ribbontail ray was made (Figures 1b and 2c). Based on morphological resemblance and a similar size (DW = 22 cm, TL = 48 cm), we deem it most likely this observation was a “recapture” of specimen one instead of a third deformed individual (Figure 2a,c). During the survey of April 8th, the deformed ray was observed digging into the sediment with its snout uplifted, a balancing behavior associated with feeding in *T. lymma* (Appendix 1) (Madduppa et al., 2020).

## 4 DISCUSSION

Here, we provide the first ever evidence for an ontogenetic deformity in the bluespotted ribbontail ray, *T. lymma*. We describe two individuals with a symmetrical deformity of the posterior pectoral disk. Both individuals had grown to a disk width of 22 cm, which is well above the 14.3 ± 2.8 cm reported for neonate bluespotted ribbontail rays (Santos Ferreira, 2013). Thus, their abnormal pectoral disk did not seem to affect their survival, despite the pivotal role of the (posterior) pectoral fin in batomorph feeding and locomotion (Blevins & Lauder, 2012; Freitas et al., 2019; Rosenberger & Westneat, 1999). This may be because, in contrast to most deformities (Ribeiro‐Prado et al., 2008), the resulting body shape of our specimens does not appear to be hydrodynamically inefficient but instead somewhat resembles the body plan of certain skate species (Last et al., 2016).

Contact with anthropogenic pollutants, poor nutrition, genetic disorders, diseases, and stunted embryonic development have all been reported as potential causes of morphological abnormalities in elasmobranchs. However, data to corroborate these hypotheses are usually lacking, so the ultimate cause of batomorph deformities often remains uncertain (Ehemann et al., 2022). The same is true for this study, as we did not have access to the specimens to obtain samples for molecular, anatomical, or physiological analysis. However, the almost perfect bilateral symmetry of the deformities and the fact we observed it in two individuals seems to indicate this abnormality has a genetic basis. Moreover, the fact that we observed two individuals, while sampling a restricted number of rays could indicate the deformed rays, were closely related. Alternatively, the alleles responsible for this deformity may be present in elevated frequencies in the local (sub)population. Chemical pollution is unlikely to be the main driver behind these deformities. While our study area is located between Rabigh (~60 km) and Jeddah (~100 km) where marine sediments were previously classified as highly polluted (Youssef & El‐Sorogy, 2016). Coastal sediments closer to our study area (<15 km) were shown to have only low‐to‐moderate levels of contamination (Ruiz‐Compean et al., 2017).

Only two other cases of deformed posterior pectoral fins have previously been reported for batomorphs (Ramaiyan & Sivakumar, 1988; Ribeiro‐Prado et al., 2008). In both cases, the posterior pectoral fin was completely cleft giving a fringe‐like appearance, which starkly contrasts the symmetrical deformity presented here. Perhaps, the most similar deformity previously reported is a Chilean eagle ray, *Myliobatis chilensis* Philippi, 1892, whose pectoral fin was symmetrically split in the middle (Valderrama‐Herrera et al., 2022). Somewhat similar are the most severe, symmetrical cases of an incomplete fusion of the pectoral fin to the head, which is relatively common in batomorphs (Bureau, 1889; Clarke, 2021; Ehemann et al., 2022; Legendre, 1935; Ribeiro‐Prado et al., 2008; Templeman, 1965; Valderrama‐Herrera et al., 2022). The prevalence of incomplete disk closures in batomorphs is likely a result of the fact that the pectoral disk develops out of two separate pectoral fins that first grow in length and width and then gradually fuse with the body (Thorson et al., 1983). However, the development of the anterior and posterior pectoral fin is underpinned by different genetic pathways (Nakamura et al., 2015). The anterior growth of the pectoral fin is controlled by a unique molecular pathway driven by expression of Fgf7 and 3′Hox genes. In contrast, the posterior region develops under the influence of Gli3, Shh, and 5′Hox genes, which are part of a highly conserved molecular pathway that is similar to the genetic underpinnings of tetrapod limb development (Nakamura et al., 2015). This may explain why ontogenetic deformities of the posterior pectoral fin, such as we describe here, are so much rarer than deformities of the anterior fin.

Finally, our study highlights the multi‐modality of UAV surveys. By providing a permanent record of the environment UAV imagery enabled us to spot these uniquely deformed rays that may otherwise have gone unnoticed, even though they inhabited a university campus.

## AUTHOR CONTRIBUTIONS

**Ioana Andreea Ciocănaru:** Investigation (lead); writing – original draft (equal); writing – review and editing (equal). **Brian Owain Nieuwenhuis:** Investigation (supporting); writing – original draft (equal); writing – review and editing (equal). **Raquel Lubambo Ostrovski:** Writing – original draft (equal); writing – review and editing (equal). **Jesse Cochran:** Validation (lead); writing – review and editing (equal). **Burton H. Jones:** Funding acquisition (lead); supervision (lead); writing – review and editing (equal).

## CONFLICT OF INTEREST STATEMENT

This article was funded by KAUST baseline research funds to BJ, BAS/1/1032‐01‐01. The authors declare no competing interests.

## Data Availability

All datasets are included in the paper's main text and appendices.
